The article "HYAL1 Is Downregulated in Idiopathic Pulmonary Fibrosis and Inhibits HFL-1 Fibroblast Proliferation When Upregulated" was published in 2020. Journal: Biomed Res Int.

# HYAL1 Is Downregulated in Idiopathic Pulmonary Fibrosis and Inhibits HFL-1 Fibroblast Proliferation When Upregulated

**DOI:** 10.1155/2020/3659451

**Published:** 2020-03-11

**Authors:** Dong Leng, Xiaoxi Huang, Jiawen Yi, Hongying Zhao, Yuhui Zhang

**Affiliations:** ^1^Clinical Laboratory, Beijing Chao-Yang Hospital, Capital Medical University, Beijing 100020, China; ^2^Medical Research Center, Beijing Chao-Yang Hospital, Capital Medical University, Beijing 100020, China; ^3^Department of Respiratory and Critical Care Medicine, Beijing Chao-Yang Hospital, Capital Medical University, Beijing 100020, China; ^4^Department of Pathology, Beijing Chao-Yang Hospital, Capital Medical University, Beijing 100020, China

## Abstract

**Background:**

Idiopathic pulmonary fibrosis (IPF), the most common interstitial lung disease, arises from transforming growth factor beta 1- (TGF*β*1-) induced aberrant fibroproliferation in response to epithelial injury. The TGF*β*1-) induced aberrant fibroproliferation in response to epithelial injury. The TGF

**Methods:**

We first performed microarray data mining of previously published gene expression datasets to identify key gene signatures in IPF lung tissues. HYAL1 expression levels in IPF and normal lung tissues were then characterized using immunohistochemistry followed by real-time quantitative reverse transcription-PCR (qRT-PCR) and western blot analysis on isolated fibroblasts from fresh lung tissues of IPF and healthy donors. A human fetal lung fibroblast HFL-1 cell line, which was used in place of primary lung fibroblasts, was used to assess the proliferative or apoptotic effects associated with lentiviral-induced HYAL1 overexpression using CCK-8 cell proliferation assay and Annexin V-APC staining. The identification of potentially associated molecular pathways was performed using microarray analysis followed by qRT-PCR and western blot analysis.

**Results:**

Lung tissue microarray data mining and immunohistochemistry revealed significantly downregulation of *HYAL1* in IPF lung tissue. However, *HYAL1* in IPF lung tissue. However, *HYAL1* in IPF lung tissue. However, *HYAL1* in IPF lung tissue. However, *β*1-) induced aberrant fibroproliferation in response to epithelial injury. The TGF*β*1-) induced aberrant fibroproliferation in response to epithelial injury. The TGF

**Conclusions:**

We showed that *HYAL1* overexpression could prevent HFL-1 fibroproliferation. Furthermore, our findings suggest that transcriptional regulators and BMP receptor signaling may be involved in HYAL1 modulation in IPF therapy.*HYAL1* in IPF lung tissue. However,

## 1. Introduction

Idiopathic pulmonary fibrosis (IPF) is the most common type of interstitial pneumonia with an annual incidence rate of approximately 10 out of 100,000 cases [1, 2]. IPF presents with a higher prevalence among men than women (ratio of 1.5-1.7 : 1) and primarily affects individuals aged 50-70 years old [1]. Typical symptoms of IPF include gas exchange disruption and respiratory failure, which inevitably leads to death within 2-5 years after diagnosis [3, 4]. As the etiology of IPF is poorly characterized [5, 6] and the only effective treatment is lung transplantation [7], there is an urgent need to elucidate the mechanism of action. Excessive extracellular matrix (ECM) accumulation, formation of fibroblast and myofibroblast foci, and excessive fibroproliferation are the hallmarks of IPF [8, 9]. The major ECM constituent, hyaluronic acid (HA), was found to be increased in IPF patients [10, 11], and its ability to promote transforming growth factor beta 1- (TGF*β*1-) mediated fibroblast proliferation [3] led to IPF pathogenesis.

Hyaluronidase 1 (HYAL1), also known as lung carcinoma protein 1 (LUCA-1), is the primary endoglycosidase that degrades HA [3, 9]. The *HYAL*1 gene resides in chromosome 3p21.3 and is associated with tumor suppression suggesting its possible role in regulating cell proliferation [12]. The role of *HYAL1* as a tumor suppressor or oncogene remains unclear [12–18] with reports of both *HYAL1* downregulation in human endometrial cancer and lung and kidney carcinomas [12, 13] and upregulation in breast, epithelial ovarian, and bladder tumors [16–18]. The overall function is believed to be tumor type or concentration dependent [19] as with prostate cancer; cell proliferation was suppressed at a high HYAL1 concentration and vice versa [19]. Further convoluting evidence explains that the role of HYAL1 in the same cancer type but different species can differ. For example, it promotes colorectal tumor progression in humans but inhibits cancer proliferation in rat models [14, 20].

Abnormal tissue damage and repair often lead to tissue fibrosis [21]. IPF is the most common lung interstitial disease, and importantly, it is irreversible [22]. Hyaluronidases have shown efficacy in lung fibrosis therapy as they can increase the number of mesenchymal stem cell-like cells and reduce collagen deposition and production [23–25]. HYAL1 and TGF*β*1 were found to play antagonistic roles: *HYAL1* overexpression in murine L929 fibroblasts inhibited TGF*β*1-mediated cell growth, while TGF*β*1 inhibited the *HYAL1*-induced tumor necrosis factor- (TNF-) mediated cytotoxicity [26]. In light of these reports, we designed this study to clarify the effect and mechanism of HYAL1 expression on lung fibroblast proliferation and apoptosis. In our previous study, utilizing microarray, we identified gene expression changes in the IPF lung tissue genetic profile compared to normal tissue [27]. In the present study, we performed further analysis of the *HYAL1* gene expression profiles that have been obtained from published data mining, immunohistochemistry on paraffin-embedded lung tissues, and real-time quantitative reverse transcription-PCR (qRT-PCR) and western blot analyses on isolated primary lung fibroblasts. We also investigated the effect of *HYAL1* overexpression on HFL-1 fibroproliferation and apoptosis. Moreover, we performed microarray and bioinformatics analysis to identify key genes that were significantly altered within corresponding signaling pathways.

## 2. Materials and Methods

### 2.1. Data Mining

Data mining of the merged microarray data from our previous study of 48 IPF lung tissues (17 from GSE24206 data and 31 GSE10667 data) and 27 healthy controls (6 routine lung volume reduction after lung transplantation from GSE24206; 15 free margins with normal lung cancer histology from GSE10667; and 6 from the GSE16538 data) was performed [27–30]. Different genes with altered profiles were selected using an unpaired *t* test (*P* < 0.0001), and the general gene expression pattern was extracted through Euclidean distance similarity metric and complete linkage algorithm-based two-way clustering method using the Cluster 3.0 and Java TreeView software (Stanford University, USA). Gene expression data of significantly altered genes were further analyzed with the supervised classification method support vector machine (SVM) algorithm, which outputs a gene expression model using multtest and kernlab packages (New York University and Rockefeller, USA). Significantly altered genes with weight coefficients above specific cutoff values (0.9 for lung tissue; 0.1 for HFL-1 fibroblasts) were selected. Next, the gene expression data which met the selection criteria were dimensionally reduced through principal component analysis (PCA), and genes with higher loading coefficient (coefficient > 0.95 for HFL-1 fibroblasts) were collected as gene signatures. The PCA was completed using the prcomp command. Principal components with cumulative proportion of 85% were subjected to Bayesian probit regression for significance analysis. All analyses were completed under the R 3.5.0 environment.

### 2.2. Ethics Statement and Tissue Specimens

Experiments and subsequent data analysis were performed with approval from the Beijing Chao-Yang Hospital Ethics Committee (2017-Science-10). The Committee waived the need to obtain informed consent from subjects whose samples were used. The IPF lung tissue samples were procured from three patients diagnosed in accordance with the criteria approved by the American Thoracic Society [31]. The healthy control lung tissue samples were obtained from one healthy donor for lung transplantation and two disease-free margins of non-small-cell lung cancer patients which showed normal histology. IPF primary lung fibroblasts were isolated from surgical lung biopsy samples from three IPF patients. Normal primary lung fibroblasts were isolated from lung transplant explants of three healthy donors. The details of all patients are summarized in Table 1.

### 2.3. Immunohistochemistry

IPF and normal human lung tissue specimens (4 *μ*m thick) were formalin-fixed and paraffin-embedded on microslides. Tissue sections were treated for 1 h at 72°C, deparaffinized in xylene for 10 min twice, and rehydrated by soaking in 100%, 95%, and 75% ethanol-water solutions for 2 min each. Antigen retrieval was performed by autoclaving the samples in preheated EDTA pH 8.0 at 100% power for 2.5 min. The tissue sections were then incubated in rabbit polyclonal anti-HYAL1 primary antibody (1 : 500; Abcam 203293, UK) at 4°C overnight, followed by incubation with HRP-labeled goat anti-rabbit IgG secondary antibody (ZSGB-BIO PV-6001, China) at room temperature for 20 min. Subsequently, the sections were stained with DAB (ZSGB-BIO ZLI-9017, China) at room temperature for 5 min and then counterstained with hematoxylin (ZSGB-BIO ZLI-9017, China) at room temperature for 20 min before examination under an optical microscope (Olympus CX31, USA). The HYAL1 expression in lung tissues by immunohistochemistry was analyzed by average integrated optical density (IOD) using Image-Pro Plus 6.0 software (Media Cybernetics, USA).

### 2.4. Primary Lung Fibroblast Cell Culture

Human lung tissues of both IPF patients and healthy donors were minced and allowed to adhere to the bottom of the culture flask. Samples were cultured for 4 h after attachment to the culture flask bottom, in Dulbecco's Modified Eagle's Medium (DMEM) supplemented with 10% (*v*/*v*) fetal bovine serum (FBS; Gibco, USA), 100 mg/mL streptomycin, and 100 U/mL penicillin at 37°C in a 5% CO_2_ humidified incubator. The cell culture medium was refreshed every 3 days, and the cells were passaged at a 1 : 2 ratio every 3 days.

### 2.5. HFL-1 Cell Culture

Human fetal lung fibroblast HFL-1 (Type Culture of the Chinese Academy of Science, Shanghai, China) cells in F-12K medium (Invitrogen, USA) supplemented with 10% (*v*/*v*) fetal bovine serum were cultured at 37°C in a 5% CO_2_ humidified incubator. The cell culture medium was replaced every 2 days, and the cells were passaged at a 1 : 2 ratio every 3 days.

### 2.6. HYAL1 Transfection into Fibroblasts

Recombinant HYAL1 plasmid was constructed using the GV492 lentivirus particle and the specific primers (GeneChem, Shanghai, China) of full-length human hyaluronidase *Hyal*1: 5′-AGGTCGACTCTAGAGGATCCCGCCACCATGGCAGC CCACCTGCTTCC-3′ (forward) and 5′-TCCTTGTAGTCCATACCCCACATGCT CTTCCGCTCACACC-3′ (reverse). The GV492 lentivirus particle, control vector CON335, and the specific primers were purchased from GeneChem (Shanghai, China). The lentivirus *Hyal*1 and the control CON 335 were transfected into 40% confluent HFL-1 fibroblasts in the presence of 5 *μ*g/mL polybrene, and thereafter, the cell culture medium was replaced 16 h postinfection.

### 2.7. Gene Expression Profiling and Data Preprocessing

Gene expression profiling of HFL-1 fibroblasts transiently infected with the lentivirus *Hyal*1 and the control were performed using GeneChip® PrimeView™ Human Gene Expression Array (Affymetrix, USA). Total RNA was extracted from cells using the Total RNA Isolation Reagent Trizol (Superfect TRI™, Shanghai, China). The RNA concentration and purity were determined using the NanoDrop 2000 (Thermo Fisher, Massachusetts, USA), and the RNA integrity was assessed using the 2100 Bioanalyzer (Agilent, California, USA). *In vitro* transcription (IVT) was then performed to obtain fragmented biotin-labeled RNA according to the manufacturer's instructions (GeneChip 3′-IVT Express Kit, Affymetrix, California, USA). Next, the fragmented biotin-labeled RNA was hybridized to the Affymetrix chip and measured with GeneChip Scanner 3000 (Thermo Fisher, Massachusetts, USA). Data were saved as .CEL files, which could be accessed through the GEO repository (http://www.ncbi.nlm.nih.gov/geo/) with the accession number GSE131443 (the data are scheduled to be released on Jun 30, 2020). We performed triplicate measurements of the test (overexpressed *HYAL1*: N5948-1, N5948-2, and N5948-3) and control (vector CON335-infected HFL-1 fibroblasts: N5949-1, N5949-2, and N5949-3) groups using the same Affymetrix chip. Genes with significantly altered expression profiles between the *HYAL1* overexpressed group and the negative control group (false discovery rate (FDR) < 0.05) were identified using empirical Bayesian linear modeling. The Benjamini-Hochberg method was employed to calculate the FDR. Supervised classification using the SVM algorithm and gene signature extraction were also performed as described in the data mining subsection.

### 2.8. Gene Annotation and Ingenuity Pathway Analysis

Gene set enrichment analysis (GSEA) was performed to identify genes with significantly altered expression profiles in HFL-1 fibroblasts with overexpressed *HYAL1* (loading coefficients < −0.95). The online software “The Database for Annotation, Visualization and Integrated Discovery (DAVID) v6.8” (https://david.ncifcrf.gov/) was employed. The gene interaction networks and the regulatory mechanism of *HYAL1* gene expression were subsequently predicted with the Ingenuity Pathway Analysis (IPA) software (Qiagen, Germany).

### 2.9. Real-Time Quantitative RT-PCR (qRT-PCR)

Total RNA extracted from primary fibroblasts or HFL-1 cells was reverse transcribed to cDNA using the M-MLV kit (Promega, USA) and oligo(dT) primers (Sangon Biotech (Shanghai) Co. Ltd., China). Next, cDNA amplification was performed using the SYBR Premix Ex Taq DNA Polymerase (Takara, Japan). The housekeeping gene human glyceraldehyde-3-phosphate dehydrogenase (GAPDH) was used as the internal control. The sequences of the primers used in RT-qPCR are shown in Table 2. qRT-PCR was performed using the Roche Light Cycler 480II (Switzerland), and the gene expression levels were normalized with reference to *GAPDH* using the Cq method [32].

### 2.10. CCK8 Cell Proliferation and Apoptosis Assays

Cell proliferation was assessed using the Cell Counting Kit-8 (CCK8) assay (Sigma, USA) according to the manufacturer's instructions. Infected HFL-1 fibroblasts (100 *μ*L; 2 × 10^3^ cells/well) collected at the logarithmic phase were seeded in 96-well plates and then incubated for 1, 2, 3, 4, and 5 days. Triplicate measurements of the absorbance readings were performed at 450 nm daily for the tested duration. Apoptotic HFL-1 fibroblasts infected with lentivirus carrying either recombinant HYAL1 plasmid or empty vector control were detected with Annexin V-APC (eBioscience, USA) and flow cytometry (Millipore, USA).

### 2.11. Western Blot Analysis

Primary lung fibroblasts and HFL-1 cells were harvested and lysed in 1 mM PMSF (Sigma Aldrich, Missouri, USA) RIPA (Thermo Fisher Scientific, Massachusetts, USA) lysis buffer for 30 min at 4°C, then centrifuged at 15,000 g for 10 min at 4°C. The BCA assay (Pierce, Rockford, IL, USA) was used to determine protein concentration of the lysates before 10% SDS-PAGE electrophoresis. Separated protein samples were transferred onto PVDF membrane (Millipore, Bedford, MA, USA) and incubated with primary antibodies HYAL1 (ab 203293, Abcam, Cambridge, UK), TGFBR2 (ab61213, Abcam, Cambridge, UK), BMPR2 (14376-1-AP, ProteinTech, Chicago, USA), and SMAD1/5/9 (ab66737, Abcam, Cambridge, UK) at 4°C for 2 h. The membrane was then washed and incubated with HRP-labeled secondary antibody (bs-40295G-HRP, Bioss, Beijing, China) and developed by an electrochemiluminescence solution (P0018S-2, Beyotime, Shanghai, China). Images were scanned using the Odyssey Imaging System (LI-COR Odyssey, USA) and analyzed using ImageJ software (National Institutes of Health, USA).

## 3. Results

### 3.1. HYAL1 Is a Key Signature Gene That Is Significantly Downregulated in IPF Lung Tissue

In this study, we applied SVM and PCA methods to the normalized microarray data obtained from our previous study [27] to extract key gene signatures in IPF lung tissue from controls. We identified 413 key gene signatures (weight coefficients > 0.9), and they were divided into IPF and control lung tissue groups according to gene expression estimates (data not shown). Compared with our previous study, PCA identified three additional outliers: “Advanced IPF explant lower lobe rep146” samples from GSE24206 and “UIP biological rep22” and “AEx biological rep5” samples from GSE10667. Furthermore, 229 key gene signatures (loading coefficient > 0.7) were identified and perfectly distinguished 35 IPF from 20 control lung tissue samples (data not shown). From the two-way clustering heat map (Figure 1(a)), we identified the top 50 key gene signatures (25 highest positive loading coefficients and 25 highest negative loading coefficients). *HYAL1* was among the top 25 negative key gene signatures with an SVM weight of 0.937 and PCA loading coefficient of -0.696. Significantly reduced *HYAL1* expression was noted in IPF lung tissues compared with healthy controls (*P* < 0.000001; unpaired *t* test; Figure 1(b)).

### 3.2. HYAL1 Expression Was Inhibited in IPF Lung Tissues While Upregulated in IPF Fibroblasts at the mRNA Level Only

For formalin-fixed and paraffin-embedded lung tissues, HYAL1 was predominantly expressed in the pulmonary alveoli type II alveolar cells of the negative control paracarcinoma tissue or healthy donor lung tissue (Figure 2(a)). In contrast, when fibroblast accumulation occurred in the IPF lung tissue, HYAL1 expression in the alveolar cells and in the accumulated fibroblasts was significantly reduced (Figure 2(b)). Healthy lung tissues were mainly composed of intact alveolar epithelial cells and few lung fibroblasts, unlike in IPF lung tissues where the main components were accumulated lung fibroblasts and few intact alveolar epithelial cells. The average IOD of HYAL1 in IPF was decreased compared to normal lung tissues (*P* < 0.05; unpaired *t* test; Figure 2(c)). HYAL1 expression levels in IPF and healthy lung tissues typically depend upon cell types. When compared with fibroblasts from healthy lung tissues, HYAL1 was significantly upregulated in IPF lung fibroblasts at the mRNA level (*P* < 0.05; unpaired *t* test; Figure 3(a)) but not at the protein level (*P* > 0.05; unpaired *t* test; Figure 3(b)).

### 3.3. HYAL1 Inhibits Fibroproliferation but Has No Effect on Apoptosis in HFL-1 Fibroblasts Overexpressing HYAL1

The HYAL1 mRNA level in *HYAL1*-overexpressing HFL-1 fibroblasts (*n* = 3) was upregulated approximately 177-fold compared to the negative controls (*n* = 3) (*P* < 0.01; unpaired *t* test; Figure 4(a)). The CCK8 assay revealed a 1.19-fold decrease in cell proliferation in *HYAL1* overexpressed HFL-1 fibroblasts (*n* = 3) compared to the control group (*n* = 3) (*P* < 0.001; unpaired *t* test; Figure 4(b)). However, Annexin V-APC staining showed no significant change in the apoptotic rate of *HYAL1*-overexpressing HFL-1 fibroblasts (*n* = 3) when compared to the negative controls (*n* = 3) (*P* > 0.05; unpaired *t* test; Figure 4(c)).

### 3.4. HYAL1 Upregulation Induces Alteration in Gene Expression in HFL-1 Fibroblasts

A total of 1,664 differentially expressed genes (953 upregulated and 711 downregulated) were identified in HFL-1 fibroblasts (FDR < 0.05; Figure 5(a) and [Supplementary-material supplementary-material-1]): 11 genes were noted to have up to a 1.5-fold change in gene expression level. Of these 1,664 genes, 888 key gene signatures showed weight greater than 0.1 (Figure 5(b)). Of the 888 gene signatures, 339 possessed loading coefficients greater than 0.95 (Figure 5(c)), and 90 genes were transcriptionally silent. All gene lists in each analysis are shown in [Supplementary-material supplementary-material-1].

### 3.5. Inhibition of Transcription Factor Expression in HFL-1 Fibroblasts Overexpressing HYAL1

The GSEA by DAVID revealed 90 transcriptionally silent signature genes in HFL-1 fibroblasts with overexpressed *HYAL1* and suggested that they may have DNA binding- and transcription regulation-related characteristics (*P* < 0.05; [Supplementary-material supplementary-material-1]). We identified seven downregulated genes that matched the term “GO:0045892~negative regulation of transcription, DNA-templated” from the microarray data by Empirical Bayesian linear modeling: RUNX1T1 and TRIM24 (*P* < 0.01); TBX3, TWIST1 and TWIST2 (*P* < 0.0001); and KHDRBS1 and DACH1 (*P* < 0.000001). Next, we validated these 7 identified genes with real-time qPCR using the unpaired *t* test and noted upregulation of HYAL1 (*P* < 0.01; unpaired *t* test) and downregulation of RUNX1T1 (*P* < 0.05; unpaired *t* test), TRIM24, TBX3, KHDRBS1, and DACH1 (*P* < 0.01; unpaired *t* test), while no change in gene expression level was observed for both TWIST1 and TWIST2 (*P* > 0.05; unpaired *t* test; Figure 6 and Table 3).

### 3.6. HYAL1 Upregulation in HFL-1 Fibroblasts Regulates Signaling Pathways

The identified key signature genes (FDR < 0.05, Benjamini-Hochberg method) in HFL-1 fibroblasts overexpressing *HYAL1* in this study may regulate multiple classical signal transduction pathways (Figure 7(a)). In the top 10 pathways that are predicted to be altered due to *HYAL1* overexpression, the “Osteoarthritis Pathway” was significantly inactivated (*Z*‐score<−6), and “HMGB1 (high-mobility group box 1) signaling” and “Endocannabinoid Cancer Inhibitory Pathway” were significantly activated (*Z*-score of approximately +5). Of note, the classical “Osteoarthritis Pathway” was the top signaling pathway affected by *HYAL1* overexpression. Moreover, several genes with significantly altered expression levels (Figure 7(b)) may be components of signaling pathways, such as membrane receptors (TGF*β*R2: upregulated 1.078-fold, FDR < 0.01, Benjamini-Hochberg method; BMPR2: downregulated 1.064-fold, FDR < 0.05, Benjamini-Hochberg method), nuclear transcription factors (RUNX2: downregulated 1.185-fold, FDR < 0.01, Benjamini-Hochberg method; SOX9: downregulated 1.160-fold, FDR < 0.01, Benjamini-Hochberg method; FOXO3A: upregulated 1.073-fold, FDR < 0.05, Benjamini-Hochberg method), and downstream products (ADAMTS5: upregulated 1.286-fold, FDR < 0.01, Benjamini-Hochberg method; VEGF: downregulated 1.124-fold, FDR < 0.05, Benjamini-Hochberg method; osteopontin known as SPP1: downregulated 1.221-fold, FDR < 0.05, Benjamini-Hochberg method).

The expression of TGF*β*R2 and BMPR2, as well as the downstream regulators SMAD1/5/9, was measured at the protein level. Compared to negative controls, HYAL1-overexpressing HFL-1 fibroblasts showed a 1.307-fold increase for BMPR2 (*P* < 0.05, unpaired *t* test), a 1.189-fold increase for SMAD1/5/9 (*P* < 0.05, unpaired *t* test), and a 1.027-fold increase for TGF*β*R2 (*P* > 0.05, unpaired *t* test) (Figures 8(a) and 8(b)).

IPA analysis revealed that the 36 key gene signatures in *HYAL1*-overexpressed HFL-1 fibroblasts can be organized and grouped into an interaction network with the downregulated transcription regulator SMARCA4 (SWI/SNF-related, matrix-associated, actin-dependent regulator of chromatin, subfamily a, member 4; also known as transcription activator BRG1) as the central node (*P* < 0.001; Figure 9(a)). This was validated with real-time qRT-PCR (*P* < 0.01; Figure 9(b) and Table 3).

## 4. Discussion

The role of hyaluronidases in lung fibrosis is evident from the noted therapeutic applications [33] and antifibrotic effects in bleomycin-induced lung fibrosis in mice [34]. In addition, HYAL2 was found to regulate the splicing of CD44 pre-mRNA, which determines the antifibrotic phenotype [35]. Together, these previous reports provided the motivation for our investigation into the mechanistic role of hyaluronidase in pulmonary fibrosis. Furthering our interest, HYAL1 and HYAL2 were previously reported as dual blocking agents for TGF*β*1-enhanced cell growth in murine L929 fibroblasts [26]. As the antifibrotic effects of hyaluronidases in humans are largely unknown, we compared the gene expression profiles of IPF and control lung tissues. HYAL1 expression was specifically measured in lung tissues and isolated lung fibroblasts. HYAL1 inhibitory effects and its induced gene signatures as well as the corresponding signaling pathways were measured using *HYAL1*-overexpressed HFL-1 fibroblasts.

Through previous data mining with SVM and PCA methods, we identified three IPF lung tissue sample outliers from 38 IPF and 20 control clusters [27]. In this study, clustering validation of 35 IPF (the three outlier IPF clusters were omitted) and 20 control samples was performed using the top 25 positive and 25 negative key gene signatures to evaluate the goodness of a cluster. Consistent with our previous study [27], no sample type preference was identified. HYAL1 was one of the top 25 genes that was significantly downregulated in IPF lung tissues, which supports the reported antifibrotic effect of hyaluronidases in lung fibrosis [34, 36].

Our observation of reduced HYAL1 expression in IPF lung tissue was consistent with reports of the absence of HYAL1 mRNA in lung carcinoma cell lines [12] and reduced HYAL1 protein levels in endometrial carcinomas [13]. Given the similarities between IPF and cancers [37, 38], HYAL1 downregulation in IPF may lead to malignancy. Moreover, HYAL1 expression level could potentially be a biomarker of IPF pathogenesis.

HYAL1 expression was reduced in IPF lung tissues; however, an upregulation in IPF fibroblasts was noted at the mRNA level, but not at the protein level. The conflicting results could probably be due to reduced alveolar epithelial cells in IPF lung tissue, which is the cell type that predominantly expresses HYAL1. Hence, despite upregulated HYAL1 mRNA in IPF fibroblasts, as well as the accumulation of fibroblasts, these could not alter HYAL1 downregulation in IPF lung tissue. In the present study, we used HFL-1 cells to mimic the mechanism of HYAL1-mediated regulation of fibroblast proliferation or apoptosis in primary lung fibroblasts.

Overexpression of *HYAL1* and *HYAL*2 enhanced TNF cytotoxicity and ultimately reversed TGF*β*1 effects in murine normal lung fibroblast cell line L929 [26]. This was consistent with our observations of inhibited fibroproliferation in *HYAL1*-overexpressed HFL-1 cells. The regulatory effects of *HYAL2* on gene splicing [35] also indicate the potential role of *HYAL1* in modulating gene expression as well as signaling pathways in lung fibroblasts. Future studies should focus on characterizing the effect of HYAL1 on IPF lung fibroproliferation. In contrast, hyaluronan synthases (HASs) that produce HA in response to tissue injury promote severe lung fibrosis [39]. HAS2, the major isoform that controls HA production, has been reported as upregulated in IPF fibroblasts [21]. HA fragments stimulate TGF*β*-mediated oral mucosal fibroblast proliferation [40]. HYAL1 downregulation in IPF lung tissues in this study indicated the antagonistic actions of HYAL1 and HAS2. Therefore, *HYAL1* could potentially affect the pathogenesis of lung fibrosis through counteracting HASs. Future investigations of the exact mechanism of HYAL1-mediated regulation of fibroproliferation through HA would clarify the role of HYAL1 in modulating ECM in IPF.

*HYAL1*-overexpressed HFL-1 fibroblasts were engineered to elucidate the mechanism of HYAL1-mediated regulation of signaling pathways in lung fibroblasts. Microarray analysis and data mining revealed genes with significantly altered expression levels in *HYAL1*-overexpressed HFL-1 fibroblasts compared with the normal control tissue. In addition, we identified genes that were likely inhibited by *HYAL1*overexpression. Of note, seven transcription regulators were annotated and clustered in the term group of negative transcription regulation, and five of the seven identified factors were validated by real-time qRT-PCR: Dachshund 1 (DACH1), TRIM24, TBX3, KHDRBS1, and RUNX1 translocation partner 1 (RUNX1T1). Of these five transcription regulators, DACH1, a DNA-binding transcription factor that regulates gene expression and cell fate, showed the greatest decrease in expression (fold change (FC) = −2.088; *P* < 0.01; unpaired *t* test). DACH1 expression exhibits cancer-type dependency wherein it was found to be downregulated in lung adenocarcinoma [41] but upregulated in ovarian cancer [42]. DACH1 inhibits lung cancer through binding to the p53 gene [43]. As *HYAL1* was reported to have no effect on p53-mediated cell death [26], our finding suggests a novel and indirect association between *HYAL1* and p53 through DACH1 regulation. TRIM24, TBX3, and KHDRBS1 were upregulated in lung cancer [44–46]. Hence, we noted their significant downregulation in *HYAL1*-overexpressed HFL-1 cells, which is consistent with their role in inducing fibroproliferation. The association between RUNX1T1 and lung cancer is unclear, but its binding partner RUNX1 was overexpressed in non-small-cell lung cancer [47]. Hence, HYAL1-induced inhibition of lung fibroblast proliferation may occur through the downregulation of these transcription regulators.

Of note, IPA analysis predicted that the transcription factor SMARCA4 could be a central node in the gene interaction network in *HYAL1*-overexpressed HFL-1 fibroblasts. SMARCA4 had a 1.102-fold downregulation in our microarray data (FDR < 0.01; Benjamini-Hochberg method), which was further confirmed using qRT-PCR to be a 1.550-fold downregulation (*P* < 0.01; unpaired *t* test). Further investigation demonstrated that SMARCA4 played important roles in cell proliferation as evident from its upregulation in human IPF lung tissue [48, 49] and its downregulation in adenocarcinoma NCI-H522 cells [50]. SMARCA4 could potentially regulate cell proliferation at the transcriptional level through chromatin remodeling [51, 52]. SMARCA4 downregulation and relative position as the central node in the network suggests its potential in inhibiting lung fibroblast proliferation downstream of *HYAL1*. Future studies on SMARCA4 expression including the overall effect on fibroblast proliferation should be performed to elucidate the mechanistic role in HYAL1-mediated inhibition of fibroblast proliferation. These prescribed finding will aid in obtaining new insights into the effect of hyaluronidases in IPF therapy.

From the bioinformatics analyses in the present study, the key gene signatures were predicted to be predominantly associated with the classical “Osteoarthritis Pathway.” Comparing the microarray data of *HYAL1*-overexpressed *vs.* control HFL-1 fibroblasts, we observed significant downregulation of RUNX2 (FC = −1.185, FDR < 0.01; Benjamini-Hochberg method), a transcription factor reported to be overexpressed in lung fibroblasts of non-small-cell lung cancer [53]. RUNX2 downregulation, in turn, led to VEGFA (FC = −1.124, FDR < 0.05; Benjamini-Hochberg method)/VEGFB (FC = −1.106, FDR < 0.05; Benjamini-Hochberg method) downregulation in *HYAL1*-overexpressed fibroblasts, suggesting the association between RUNX2 and HYAL1-induced inhibition of fibroblast proliferation.

Previous reports [54–56] have shown that the BMPR2 (bone morphogenetic protein receptor 2, a member of the TGF*β*R superfamily) level decreased, while its antagonist, GREM1, expression level increased, and that TGF*β*R was downregulated in IPF. From the microarray data analysis, we observed downregulated BMPR2 (FC = −1.064, FDR < 0.05; Benjamini-Hochberg method), upregulated GREM1 expression (FC = 1.124, FDR < 0.001; Benjamini-Hochberg method), and increased TGF*β*R2 levels (FC = 1.078, FDR < 0.01; Benjamini-Hochberg method) in *HYAL1*-overexpressed HFL-1 fibroblasts. The TGF*β* signaling pathway plays a central role in IPF pathogenesis, especially in regulating proliferation of lung fibroblasts during disease development [6, 57]. However, our microarray data showed very modest gene expression alterations. This is likely due to false positives from the gene expression profiling technique employed in this study [58]. We performed western blot analysis to determine the expression patterns of TGF*β*R2/BMPR2/SMAD1/5/9 (SMAD9 also known as SMAD8) proteins of the BMPR2/TGF*β*R2 signaling pathways. Significantly upregulated BMPR2 and SMAD1/5/9 protein levels were found, but no significant change in TGF*β*R2 protein level in HYAL1-overexpressed HFL-1 cells was noted. BMPR2 is a key regulator of cell proliferation [59] and could reportedly inhibit TGF*β* signaling. BMPR2 can bind BMP ligands by associating with BMPR1A, thereby leading to the phosphorylation of SMADs 1/5/9 that suppress TGF*β* signaling [60]. Thus, these results suggest that overexpressing HYAL1 in lung fibroblasts could enhance the expression of BMPR2 and the subsequent downstream signaling mediators SMAD1/5/9, which in turn suppress TGF*β* signaling, and inhibit fibroproliferation.

## 5. Conclusions

This is the first study demonstrating the association between HYAL1 and IPF and the negative correlation between *HYAL1* overexpression and HFL-1 fibroproliferation. In addition, our findings suggest that *HYAL1*-induced inhibition of fibroblast proliferation may involve changes in transcription factor levels as well as BMPR2 signaling.

## Figures and Tables

**Figure 1:** Human lung tissue gene expression. (a) Heat map of the top 50 gene signatures in the selected lung tissues of IPF (*n* = 35) *vs.* control (*n* = 20) from merged gene expression profiling data of GSE24206, GSE10667, and GSE16538. Samples were selected by two-way clustering, and gene signatures were filtered by unpaired *t* test, SVM and PCA methods. Red, green, and black pixels indicate high, low, and medium expression levels, respectively. Sample details were summarized in the supplementary file [Supplementary-material supplementary-material-1]. (b) Box plot showing the relative HYAL1 gene expression levels in IPF lung tissue (*n* = 35) *vs.* healthy control (*n* = 20; *P* < 0.000001).The *P* values were calculated using the unpaired *t* test.

**Figure 2:** HYAL1 localization in normal and IPF lung tissues. (a) Images of healthy donor lung tissues and normal tissues from disease-free margins in non-small-cell lung tissue showing high HYAL1 expression; (b) images of IPF lung tissues showing low HYAL1 expression. The average IOD of IPF lung tissues (*n* = 3) was significantly lower than that of healthy controls (*n* = 3) (*P* < 0.05). The *P* values were calculated using the unpaired *t* test. HYAL1 is stained brown (DAB staining), and nuclei are stained blue (hematoxylin staining). The scale bars for the respective images are shown at the lower left corner of each image. (c) The average IOD of HYAL1 expression in IPF lung tissues (*n* = 3) was significantly lower than that in normal controls (*n* = 3) (*P* < 0.05). The *P* values were calculated using the unpaired *t* test. ^∗^*P* < 0.05.

**Figure 3:** qRT-PCR and western blot analyses of HYAL1 in normal and IPF primary lung fibroblasts. (a) Relative mRNA levels of HYAL1 in normal and IPF primary lung fibroblasts. Control: normal lung fibroblasts (*n* = 3); IPF: IPF lung fibroblasts (*n* = 3). (b) Western blot of HYAL1 in normal and IPF primary lung fibroblasts. (b1) Relative protein levels of HYAL1 in normal (*n* = 3) and IPF (*n* = 3) primary lung fibroblasts; (b2) western blot of HYAL1 and GAPDH in normal and IPF primary lung fibroblasts. All *P* values were calculated using the unpaired *t* test. ^∗^*P* < 0.05.

**Figure 4:** qRT-PCR profile of HYAL1 in *HYAL1*-overexpressed HFL-1 fibroblasts, HFL-1 fibroblast proliferation, and apoptosis. (a) NC: HFL-1 fibroblasts infected with lentivirus containing CON335 empty vector (*n* = 3); OE: HFL-1 fibroblasts infected with lentivirus containing *HYAL1* recombinant plasmid (*n* = 3). (b) CCK-8 assay cell viability plot of HYAL1-overexpressed (HYAL1) and control (CON335) HFL-1 fibroblasts (*n* = 3; mean ± SD). (c) Plot showing Annexin V staining of apoptotic cells in HYAL1-overexpressed (HYAL1) and control (CON335) HFL-1 fibroblasts (*n* = 3; mean ± SD). All *P* values were calculated using the unpaired *t* test. ^∗^*P* < 0.05; ^∗∗^*P* < 0.01.

**Figure 5:** Two-way clustering heat maps of HFL-1 fibroblasts. Heat maps showing genes with significantly altered expression levels with (a) FDR < 0.05 analyzed using the unpaired *t* test, (b) weight > 0.1 analyzed using the SVM method, and (c) loading coefficient > 0.95 analyzed using the PCA method. Red, green, and black pixels represent high, low, and medium expression levels, respectively. NC: HFL-1 fibroblasts infected with CON335 empty vector lentivirus (*n* = 3); OE: HFL-1 fibroblasts infected with lentivirus carrying *HYAL1* recombinant plasmid (*n* = 3). The detailed gene lists in each heat map are shown in [Supplementary-material supplementary-material-1].

**Figure 6:** qRT-PCR profiles showing the relative mRNA levels of genes in *HYAL1*-overexpressing HFL-1 fibroblasts and the controls. NC: HFL-1 fibroblasts infected with lentivirus containing CON335 empty vector (*n* = 3); OE: HFL-1 fibroblasts infected with lentivirus containing *HYAL1* recombinant plasmid (*n* = 3). The *P* values were calculated using the unpaired *t* test. ^∗^*P* < 0.05; ^∗∗^*P* < 0.01.

**Figure 7:** Potential gene expression regulatory modes of *HYAL1*-overexpressed HFL-1 fibroblasts. (a) IPA clustering of classical signaling pathways that are regulated by all 1,664 genes with significantly altered expression profiles (FDR < 0.05; Benjamini-Hochberg method) in *HYAL1*-overexpressed HFL-1 fibroblasts. Negative and positive *Z*-scores are represented by blue and orange, respectively. A *Z*‐score < −2 indicates a strongly inhibited gene while a *Z*‐score > 2 indicates a strongly activated gene. (b) Genes with significantly altered expression levels (highlighted) along with other associated molecules are mapped to the classical osteoarthritis pathway. Upregulated and downregulated molecules are represented in red and green, respectively, and the different shades of color correspond to the different degree of regulation.

**Figure 8:** Western blot analysis of TGF*β*R2, BMPR2, and SMAD1/5/9 in negative controls and HYAL1-overexpressing HFL-1 fibroblasts. (a) Western blot of TGF*β*R2, BMPR2, and SMAD1/5/9 in negative controls (*n* = 3) and HYAL1-overexpressing HFL-1 fibroblasts (*n* = 3); NC: HFL-1 fibroblasts infected with lentivirus containing CON335 empty vector (3 independent replicates); OE: HFL-1 fibroblasts infected with lentivirus containing *HYAL1* recombinant plasmid (3 independent replicates). (b) Relative protein levels of TGF*β*R2, BMPR2, and SMAD1/5/9 in negative controls (*n* = 3) and HYAL1-overexpressing HFL-1 fibroblasts (*n* = 3); NC: HFL-1 fibroblasts infected with lentivirus containing CON335 empty vector (3 independent replicates); OE: HFL-1 fibroblasts infected with lentivirus containing *HYAL1* recombinant plasmid (3 independent replicates). All *P* values were calculated using the unpaired *t* test. ^∗^*P* < 0.05.

**Figure 9:** SMARCA4 gene in HYAL1-expressed HFL-1 fibroblast is found in the central node in the IPA gene interaction network analysis. (a) Gene interaction networks of significantly altered genes from IPA analysis. Upregulated and downregulated molecules are represented in red and green, respectively. The different shades of colors correspond to varying extent of regulation. Solid lines represent direct interactions, solid lines with arrows represent direct activations, and dashed lines represent indirect interactions. (b) qRT-PCR profile of SMARCA4 in *HYAL1*-overexpressing HFL-1 fibroblasts and the controls. NC: HFL-1 fibroblasts infected with lentivirus containing CON335 empty vector (*n* = 3); OE: HFL-1 fibroblasts infected with lentivirus containing *HYAL1* recombinant plasmid (*n* = 3). All *P* values were calculated using the unpaired *t* test. ^∗∗^*P* < 0.01.

**Table 1:** General information of tissues and lung fibroblasts obtained from test subjects.

Sample number	Sample source	Sample type	Age (years old)	Gender
A1	Disease-free margins of non-small-cell lung cancer	Lung tissue	47	F
A2	Lung transplant explant of healthy donor	Lung tissue	Unknown	Unknown
A3	Disease-free margins of non-small-cell lung cancer	Lung tissue	68	F
Control4	Lung transplant explant of healthy donor	Lung primary fibroblast	Unknown	Unknown
Control5	Lung transplant explant of healthy donor	Lung primary fibroblast	Unknown	Unknown
Control6	Lung transplant explant of healthy donor	Lung primary fibroblast	Unknown	Unknown
B1	Surgical lung biopsy of IPF	Lung tissue	61	M
B2	Surgical lung biopsy of IPF	Lung tissue	56	M
B3	Surgical lung biopsy of IPF	Lung tissue	66	M
IPF4	Surgical lung biopsy of IPF	Lung primary fibroblast	61	M
IPF5	Surgical lung biopsy of IPF	Lung primary fibroblast	55	M
IPF6	Surgical lung biopsy of IPF	Lung primary fibroblast	58	M

**Table 2:** Primer sequences used for real-time qRT-PCR.

Gene symbol	Forward primer sequence (5′ to 3′)	Reverse primer sequence (5′ to 3′)	PCR product (bp)
HYAL1	CGATATGGCCCAAGGCTTTAG	ACCACATCGAAGACACTGACAT	129
GAPDH	TGACTTCAACAGCGACACCCA	CACCCTGTTGCTGTAGCCAAA	121
KHDRBS1	CTCCAGCACCAAGAGCACG	CTGGTCCCATTCCAGTCGT	235
TBX3	TGAACTCAACAGCCGCTCCTC	CTTCCAAGCCGCTAACCAACC	128
RUNX1T1	ACCCGAGATAGGAGAAAGA	AAAGGTCTCAGTGGGAAGT	117
DACH1	ATGTGGAACAAGTTCGCATCC	TGCAGTCATTGTAGAGGGTCT	108
TRIM24	CAGCCACAAATGCCTAAGCAG	GTGTTGGGAACTTGGATAACTGG	94
TWIST2	AAAGGCGAATCCACTCATAC	AATGATAGAGTCAGCACCAGAG	110
TWIST1	GTCCGCAGTCTTACGAGGAG	GCTTGAGGGTCTGAATCTTGCT	156
SMARCA4	TGAGAATGCCAAGCAAGATG	AGGATGCCGTTCAGGTTGT	210

**Table 3:** Real-time qRT-PCR results of *HYAL1* and eight transcription factors.

Gene symbol	Gene full name	Molecular type	Fold change	*P* value
HYAL1	Hyaluronidase 1	Enzyme	177.453	0.0033
KHDRBS1	KH RNA binding domain containing, signal transduction associated 1	Transcription regulator	-1.724	0.0019
TBX3	T-box 3	Transcription regulator	-1.433	0.0016
RUNX1T1	RUNX1 translocation partner 1	Transcription regulator	-1.435	0.0217
DACH1	Dachshund family transcription factor 1	Transcription regulator	-2.088	0.0010
TRIM24	Tripartite motif containing 24	Transcription regulator	-1.245	0.0038
TWIST2	Twist family bHLH transcription factor 2	Transcription regulator	-1.156	0.1599
TWIST1	Twist family bHLH transcription factor 1	Transcription regulator	-1.130	0.2024
SMARCA4	SWI/SNF related, matrix associated, actin dependent regulator of chromatin, subfamily a, member 4	Transcription regulator	-1.550	0.0089

## Data Availability

The datasets generated and analyzed during the current study are available from the corresponding author on reasonable request.

## Supplementary Materials

Supplementary 1 Table S1: gene expression data of differentially expressed genes for lentiviral-induced HYAL1 overexpressed HFL-1 and controls.

Supplementary 2 Table S2: gene lists and corresponding parameters in three analyses.

Supplementary 3 Table S3: DAVID gene ontology functional annotation chart of 90 silent signature genes in HYAL1-overexpressed HFL-1 fibroblasts.

Supplementary 4 Table S4: sample details for GEO data mining.
